The article "Antioxidant Activity, Polyphenolic Content, and FT-NIR Analysis of Different Aspilia africana Medicinal Plant Tissues" was published in 2021. Journal: Evid Based Complement Alternat Med.

# Antioxidant Activity, Polyphenolic Content, and FT-NIR Analysis of Different *Aspilia africana* Medicinal Plant Tissues

**DOI:** 10.1155/2021/9917810

**Published:** 2021-09-14

**Authors:** Denis Okello, Yuseong Chung, Hyoseon Kim, Jun Lee, Endang Rahmat, Richard Komakech, Yong-Goo Kim, Francis Omujal, Youngmin Kang

**Affiliations:** ^1^Herbal Medicine Resources Research Center, Korea Institute of Oriental Medicine (KIOM), 111 Geonjae-ro, Naju-si, Jeollanam-do 58245, Republic of Korea; ^2^Korean Convergence Medicine Major, University of Science and Technology (UST), Daejeon, Republic of Korea; ^3^Gombe Secondary School, P.O. Box 192, Butambala, Mpigi, Uganda; ^4^Natural Chemotherapeutics Research Institute (NCRI), Ministry of Health, P.O. Box 4864, Kampala, Uganda

## Abstract

*Aspilia africana* has been used for generations to treat many diseases in Africa. Its biological activities, including antioxidant and anti-inflammatory potential, are attributed to a number of secondary metabolites, including alkaloids and polyphenolics. The antioxidant activities of *A. africana* callus (CA), juvenile *in vitro* leaf (IL) and root (IR), *ex vitro* root (SR) and leaf (SL), and wild leaf (WL) dried samples were assessed based on their diphenylpicrylhydrazyl (DPPH) free radical scavenging abilities. The total phenolic and flavonoid content of different plant samples was compared. Further, high-pressure liquid chromatography (HPLC) was used to quantitatively determine chlorogenic acid content in the *A. africana* plant samples. Fourier transform near-infrared (FT-NIR) analysis was also carried out to compare the antioxidant phytochemical content in the *A. africana* plant tissues. Among the samples, IR, with the highest total phenolic content (167.84 ± 1.057 mg GAE/g), total flavonoid content (135.06 ± 0.786 mg RUE/g), and chlorogenic acid (5.23 ± 0.298 mg/g) content, had the most potent antioxidant activity (IC_50_ = 27.25 ± 5.028 *μ*g/mL), followed by WL. The lowest polyphenolic content and antioxidant activity were observed in SR. The antioxidant activities of *A. africana* tissues were positively correlated with the total phenolic and flavonoid content in the samples. The differences in antioxidant activities of *A. africana* tissues could be attributed to the difference in their polyphenolic content. Our study reports, for the first time, the antioxidant activities of *A. africana* callus and roots (*in vitro* and *ex vitro*). The *A. africana* samples IR, CA, and WL could be valuable natural sources of antioxidants that could be further exploited for the development of useful pharmaceutical products.

## 1. Introduction

Redox processes that occur during metabolism in aerobic cells generate reactive oxygen and nitrogen species at low or moderate concentrations. These species possess important physiological functions, including transduction of cellular signals and defense against pathogens [1, 2]. If these reactive species are not regulated, they attack vital biological molecules such as proteins, RNA, DNA, lipids, and carbohydrates, leading to cell death, tissue damage, and eventually to the development of chronic diseases [1, 3]. Antioxidants defend the body against diseases such as cancer, atherosclerosis, neurodegenerative diseases, cardio\vascular diseases, arthritis, diabetes mellitus, and nephritis [1, 4]. Plants possess powerful antioxidants, and the use of these plants in diets or as medicinal herbs reduces the occurrence of such diseases [3, 5].

The medicinal plant *Aspilia africana* (Pers.) C. D. Adams belongs to the family Asteraceae and has been used for generations to treat diseases in many African countries [6]. The plant is used to treat wounds, osteoporosis, stomachache, rheumatic pains, ear infections, tuberculosis, cough, febrile headaches, wounds, gonorrhea, measles, diabetes, diarrhea, gastric ulcers, sores, malaria, and inflammatory conditions [5–7]. The biological activities of *A. africana*, including antioxidant, anti-inflammatory, wound healing, anticancer, antidiabetic, and antiulcer activities, are mainly attributed to the polyphenolic group of compounds [6, 7]. For the traditional treatment of diseases, the commonly used plant parts of *A. africana* are leaves and roots collected from the wild [5].

Polyphenols are a large category of secondary metabolites that are abundantly present in medicinal plants and display excellent antioxidant properties [8]. These groups of chemical compounds are differentiated based on their synthetic pathways [8]. A wide and highly heterogeneous group of polyphenols, which includes phenylpropanoids, lignins, condensed tannins, and flavonoids, is derived from an L-phenylalanine precursor, and the second largest group consisting of hydrolyzable tannins is derived from a gallic acid precursor [8]. Currently, pharmacologists and researchers are interested in the phenolic and flavonoid content of plants, their antioxidant capacities, and their roles in preventing deadly diseases such as cardiovascular diseases, neurodegenerative diseases, and cancer [4]. Polyphenols possess hydroxyl (OH) groups, which act as positive moieties for their antioxidant activities [9].

Chlorogenic acid (Figure 1) is a phenylpropanoid compound produced during respiration (aerobic) in the shikimic acid pathway in plants [10]. It is a condensation product of quinic and caffeic acids and is an active ingredient in several medicinal plants [10, 11]. Although chlorogenic acid is common in plants, only a few plants have it in high concentrations [9].

Chlorogenic acid was previously detected in the most active leaf extracts of *A. africana* [12, 13]. It has been characterized as an important polyphenol in the Lamiaceae and Asteraceae families [9]. It is a well-known antioxidant [9, 14, 15] and is used in the treatment of type 2 diabetes, Alzheimer's disease, stroke, eclampsia, and obesity [14]. Further, chlorogenic acid has been shown to improve lipid metabolism and glucose tolerance [16, 17], and its antimicrobial [18, 19] and anxiolytic [19, 20] activities are well-documented. The antioxidant activity of plants such as coffee is dependent on phenolic compounds, especially its chlorogenic acid content [21]. Chlorogenic acid significantly inhibits the oxidative stress induced by interleukin-8 (IL-8) secretion and mRNA expression [9]. Additionally, IL-8 production is suppressed by caffeic acid, a metabolite of chlorogenic acid [9].

Anxiety is a psychiatric and most prevalent Central Nervous System (CNS) disorder with high comorbidity and morbidity [22]. The increase in its prevalence worldwide is due to the inhumane and highly competitive atmosphere in man's everyday life [23]. Thus, anxiolytic substances are among the most consumed drugs by humans [23]. The current anxiolytic drugs are associated with many adverse effects, including psychomotor function decay, dependence and abstinence syndromes, anterograde amnesia, and paradoxical reactions [22, 23]. Carlini [23] points out that alternative medication with fewer adverse effects could be derived from medicinal plants that have been utilized for generations to treat similar conditions. *A. africana* has been used to treat some CNS-related disorders such as epilepsy [24], and its ethanolic leaf extract was confirmed to possess sedative and antiseizure properties [25]. The sedative, antiseizure, and apparent anxiolytic potentials of the plant were attributed to its richness mainly in flavonoids [25]. Flavonoids are apparently the main active principles responsible for the sedative/anxiolytic effects of the most medicinal plant [23]. Antioxidants eliminate reactive nitrogen and oxygen species and suppress the oxidative stress pathway, therefore protecting against neuronal damage triggered by oxidative stress resulting in remission and functional recovery from symptoms of anxiety [26].

*A. africana* has been confirmed to contain polyphenolic compounds and vitamins, including ascorbic acid, riboflavin, and thiamine, which possess antioxidant activities [5, 6]. The compound parahydroxybenzaldehyde, isolated from the methanolic leaf extract of *A. africana*, competed favorably in comparison to standard antioxidant drugs [27]. There are a few studies on the antioxidant activity of *A. africana* leaves. However, to the best of our knowledge, this is the first study to determine the antioxidant activities of *A. africana* calli, and juvenile *in vitro* regenerated *A. africana* leaves and roots and to quantitatively compare total phenolic, flavonoid, and chlorogenic acid content in different plant tissues. In addition, Fourier transform near-infrared spectroscopy (FT-NIR) was performed to compare the antioxidant chemical content of *A. africana* plant tissues. Therefore, this study offers a basis for developing pharmaceutical products, including novel anxiolytic drugs, from this unique plant resource.

## 2. Materials and Methods

### 2.1. Explant Sterilization, Callus Induction, and Culture

Shoots of *A. africana* plants (100–120 mm from the tip) were excised from three-month-old plants in a smart farm at Herbal Medicine Resources Research Centre, Korea Institute of Oriental Medicine (KIOM)-Naju. The shoots were washed under running tap water for 5 min and moved to a laminar flow bench. The *A. africana* shoots were washed again with autoclaved distilled water and sterilized using 100% (v/v) and 70% (v/v) ethanol for 20 and 30 s, respectively, and in 2% (v/w) sodium hypochlorite for 3 min. Finally, the shoots were rinsed four times with sterile water.

The leaves (except the terminal leaf pairs) were excised from the shoots and cut into 7 mm^2^ segments, which were used as explants for callus induction. Nine leaf segments were placed in each Petri dish containing 3 g/L gerlite-gelled MS medium with vitamins and supplemented with benzylaminopurine (BAP, 0.5 mg/L) and 2,4-dichlorophenoxyacetic acid (2,4-D, 1.0 mg/L). Sixty replicates were made, and the Petri dishes were placed in the dark at 25 ± 2°C and relative humidity of 75% until the calli developed. The calli were subcultured twice at four-week intervals and maintained under a 16-h photoperiod with light provided by cool white fluorescent tubes at 25°C and 70% relative humidity. The calli were washed under running tap water to remove traces of the medium and then dried for 24 h in an oven at 60°C. The dried callus (CA) was homogenized into a fine powder and stored at 4°C until extraction for analysis.

### 2.2. *In Vitro* Leaf and Root Induction, Culture, and Processing

The sterile *A. africana* shoot apices were cut into 30–45 mm long pieces and end surfaces that were in contact with the sterilizing agents were removed. The shoot apices were inoculated in 3 g/L gerlite-gelled MS medium with vitamins fortified with 1-Naphthaleneacetic acid (NAA, 0.1 mg/L) for *in vitro* root induction. Four shoot apices were placed in individual 125 × 100 mm culture vessels with 100 replications and then placed under a 16 h photoperiod with light provided by cool white fluorescent tubes at 25°C and 70% relative humidity. After 6 wk, the *in vitro* leaves (IL) and roots (IR) were excised, washed, dried, homogenized, and stored in the same way as the calli, ready for analysis.

### 2.3. Leaf and Root Samples from Three-Month-Old *A. africana* Plants, Collecting, and Processing

Three-month-old *A. africana* plants grown in a greenhouse at Herbal Medicine Resources Research Centre, Korea Institute of Oriental Medicine (KIOM)-Naju were randomly chosen and carefully uprooted, and their roots were washed under running tap water. The leaves (SL) and roots (SR) were harvested and dried in an oven at 60°C for 24 h. The dried leaf and root samples were homogenized into a fine powder and stored at 4°C until extraction for analysis.

### 2.4. Wild *A. africana* Leaf Sample Collection and Processing

Leaves of wild *A. africana* plants (WL) were randomly collected from more than 50 plants in Pece, Gulu district, Uganda, East Africa. The leaves were sun-dried for 5 d, homogenized into a fine powder, packed in airtight bags, and posted to the Korea Institute of Oriental Medicine (KIOM), Herbal Medicine Resources Research Centre, Republic of South Korea. The samples were stored at 4°C until analysis.

### 2.5. Antioxidant Capacity Assay

A month after harvesting, about 2 g of each powdered sample (wild leaves, *in vitro* roots and leaves, green house roots and leaves, and callus of *A. africana*) was added to 50 mL of 80% ethanol and sonicated at 40°C for 1 h. The sample extracts were filtered (using a syringe filter with a 0.45 *μ*m pore size membrane) and the filtrate was concentrated in a rotary evaporator (EYELA N-1200B, Tokyo Rikakikai Co. Ltd., Japan) at 40°C under reduced pressure. Fifty milligrams of each concentrated *A. africana* sample (dried extract) was added to 5 mL of 80% aqueous ethanol to form a 10000 *μ*g/mL stock solution. The stock solution for each sample was diluted to varying concentrations (25, 100, 200, and 300 *μ*g/mL) for the antioxidant assay.

The antioxidant capacity of *A. africana* samples was determined using the diphenylpicrylhydrazyl (DPPH) radical scavenging method modified from Sarker and Oba [4]. To 0.1 mL solution of DPPH (Sigma-Aldrich, St. Louis, MO, USA) in ethanol, 0.1 mL of the *A. africana* sample was added at different concentrations in triplicate in a 96-well microplate, wrapped in aluminum foil, and incubated at 37°C for 30 min. Spectrophotometric measurements were performed with Spectramax i3x (Molecular Devices, Wokingham, UK) at 517 nm. The radical scavenging activity was expressed in terms of antioxidant percentage calculated from the following formula:

(1) $$\begin{array}{c} \text{antioxidant activity}\left(\%\right)=\left[\frac{A_{\text{control}}-A_{\text{sample}}}{A_{\text{control}}}\right]\times 100, \end{array}$$

where *A*_control_ = absorbance of the control sample and *A*_sample_ = absorbance of the test sample.

Gallic acid was used as a positive control in this study. The IC_50_ values (sample concentration required to scavenge 50% DPPH free radicals) were derived from a simple regression analysis. The sample extraction and DPPH antioxidant assays were carried out after storing the samples at 4°C for one month.

### 2.6. Determination of Total Polyphenolic Content

#### 2.6.1. Total Phenolic Content

The total phenolic content of the *A. africana* samples was estimated following the method of Derakhshan et al. [28], with modifications. The previously prepared stock extract of each sample was diluted to obtain 0.3 mg/mL sample, of which 0.5 mL aliquot was taken in a 1.5 mL microcentrifuge tube and mixed with the same volume of Folin-Ciocalteu's reagent. After 4 min, 0.5 mL of 10% Na_2_CO_3_ was added to the mixture, mixed thoroughly and incubated in the dark for 60 min at 25°C. Spectrophotometric measurements were performed with Spectramax i3x (Molecular Devices, Wokingham, UK) in triplicate for each sample, and absorbance was read at 725 nm. A calibration curve of standard gallic acid was constructed to determine the total phenolic content of each sample. The total phenolic content in each sample was expressed as mg gallic acid equivalent (mg GAE/g).

#### 2.6.2. Total Flavonoid Content

The method used by Lee et al. [29] was modified to determine the total flavonoid content of *A. africana* samples. In brief, 0.1 mL of each sample extract (1 mg/mL) was taken in a 1.5 mL microcentrifuge tube, and 0.8 mL diethyl glycol (90%), and 10 *μ*L of 1 N sodium hydroxide solution was added to the tube. This mixture was then vortexed for about 3 sec and incubated for 60 min in a water bath at 37°C. Spectrophotometric measurements were performed with Spectramax i3x (Molecular Devices, Wokingham, UK) in triplicate for each sample and absorbance was read at 420 nm. The total flavonoid content in each sample was determined from the calibration curve of the standard, rutin, and expressed as mg rutin equivalent (mg RUE/g).

### 2.7. Sample Preparation for HPLC Analysis and Quantification of Chlorogenic Acid

Powdered *A. africana* WL, SL, SR, IL, IR, and CA samples (0.2 g each) were extracted using 10 cm^3^ of 80% high-pressure liquid chromatography (HPLC) grade methanol for 60 min using sonication. The extract was filtered through Whatman grade 1 filter paper and the filtrate was refiltered using a syringe filter (13 mm, 0.45 *μ*m pore size PTFE membrane) for HPLC analysis. Standard chlorogenic acid (1.2 mg) was dissolved in 1 mL of 80% HPLC grade methanol to make a stock solution (1200 *μ*g/mL) and diluted to varying concentrations (120, 60, 30, 15, and 7.5 *μ*g/mL).

An HPLC system (1200 series, Agilent Technologies, Palo Alto, CA, USA) equipped with a photodiode array detector (PDA) was used for the analysis. Reversed-phase chromatography was performed in a binary mode of gradient and isocratic mobile phase with a reversed-phase C-18 column (Luna 5 *μ*m C-18(2) 100 Å, New Column 250 × 4.6 mm) at 25°C. The following running conditions were maintained: 10 *μ*L injection volume; mobile phase consisting of acetonitrile (A) and 0.1% acetic acid in water (B) was used as follows: 5% A (0 min), 5–20% A (0–15 min) and 20% A (15–50 min); flow rate: 0.7 mL/min; run time: 50 min; ultraviolet (UV) detection wavelength of 200–400 nm. Chlorogenic acid was identified by comparing the sample chromatographic peaks with the standard retention time. After the analysis, the peak areas were calculated using a Winchrom integrator. The five concentrations of chlorogenic acid (7.5, 15, 30, 60, and 120 *μ*g/mL) were subjected to regression analysis to calculate the calibration equation and correlation. The amount of chlorogenic acid in each sample was expressed as mg/g of the extract.

### 2.8. Fourier Transform Near-Infrared Spectroscopy (FT-NIR) Analysis

The analysis was performed using a TANGO FT-NIR spectrometer (Bruker Optics, Billerica, MA, USA) on the powdered WL, SL, SR, IL, IR, and CA samples. Calibration of the spectrometer was performed with a Light Trap: (Type 1002961, ECL 00) and Gold standard (Type 1024957, ECL: 01). Further, 2 g of each sample was analyzed in glass vials (22 mm). The absorbance spectra were obtained at 12487–3948 cm^−1^ wave numbers, which determined the different classes of compounds, including antioxidant constituents, in the samples based on their functional groups. Dendrograms were constructed for the samples based on Ward's clustering algorithm upon characteristic preprocessing of data (first derivative) and vector normalization and standardization of the Euclidean distance in the 9981–4014 cm^−1^ frequency range. The software OPUS TANGO-R was used for the Ward algorithm. Homogeneous categories were sorted maximally using the minimum variance method analysis of clusters.

### 2.9. Statistical Analysis

All experimental data were subjected to one-way analysis of variance (ANOVA) with Tukey's post hoc test using Prism (GraphPad software, v 5.03). All means were considered statistically significantly different at *p* ≤ 0.05.

## 3. Results

### 3.1. Callus Induction

A high rate of callus induction (87%) from the leaf segment explants in the callus induction medium was attained within 4-5 wk. The calli generated were cream to brown, friable, and structurally compact (Figure 2).

### 3.2. Antioxidant Capacity of *A. africana* Tissues

The DPPH antioxidant activity of *A. africana* samples was assessed at varying concentrations. The antioxidant activity of the *A. africana* samples was generally good, with over 50% DPPH inhibition for all samples at concentrations of 200 and 300 *μ*g/mL (Figure 3). Overall, the highest antioxidant activity was observed for IR (Figures 3 and 4). The DPPH antioxidant activity of all the tested samples increased with increasing concentrations (Figure 3). The highest DPPH free radical scavenging activity was observed for IR with values of 86.32 ± 0.592% and 88.43 ± 0.796% at a concentration of 200 and 300 mg/mL, respectively. These values did not differ significantly from those of the positive control, gallic acid, even at the highest concentration used (Figure 3). CA had the highest overall antioxidant activity after IR, with values of 82.85 ± 1.098% and 85.69 ± 0.906% DPPH inhibition at a concentration of 200 and 300 mg/mL, respectively (Figure 3).

The antioxidant activity of CA did not differ significantly from that of WL, nor did the antioxidant activity of IL differ significantly from that of SL (Figures 3 and 4). IR had the lowest IC_50_ value (27.25 ± 5.028 *μ*g/mL), confirming its good DPPH antioxidant activity. It was followed by CA and WL, whose IC_50_ values did not differ significantly (*p* < 0.05) (Figure 4). In contrast, the lowest antioxidant activity among the samples was of SR, with a significantly higher IC_50_ value (178.45 ± 1.609 *μ*g/mL) compared to the rest of the samples (Figure 4). For the positive standard, the IC_50_ value was as low as 2.62 ± 0.307 *μ*g/mL (Figure 4).

### 3.3. Total Phenolic and Flavonoid Content

The total phenolic and flavonoid content varied significantly in the *A. africana* samples (Figure 5). The total phenolic content of the *A. africana* tissues ranged from 16.77 ± 0.282 to 167.84 ± 1.057 mg GAE/g, whereas the total flavonoid content ranged from 55.92 ± 0.939 to 135.06 ± 0.786 mg RUE/g (Figure 5). The highest total phenolic and flavonoid content was observed in IR at 167.84 ± 1.057 mg GAE/g and 135.06 ± 0.786 mg RUE/g, respectively. These values were significantly higher than the values of WL, which possessed the second-highest total phenolic (149.98 ± 1.032 mg GAE/g) and flavonoid (97.98 ± 0.749 mg RUE/g) content (Figure 5) among the samples. Among the samples, the lowest total phenolic and flavonoid content was observed in SR at 55.92 ± 0.939 mg GAE/g and 33.41 ± 2.351 mg RUE/g, respectively (Figure 5).

### 3.4. Chlorogenic Acid Content of *A. africana* Tissues

Chlorogenic acid in the *A. africana* samples was identified by comparing the HPLC retention time, UV absorption, and mass spectra with those of the chlorogenic acid standard (Figure 6). Chlorogenic acid was detected in all the samples analyzed, as shown in the HPLC chromatograms in Figure 6.

A quantitative assessment of chlorogenic acid was performed at 280 nm. The highest quantity of chlorogenic acid was observed in IR at 5.23 ± 0.298 mg/g. This value was significantly higher (*p* < 0.05) than that in the rest of *the A. africana* samples analyzed, except in SL (4.308 ± 0.394 mg/g) (Figure 7). The chlorogenic acid content in WL, IL, SA, and CA did not differ significantly (Figure 7). The lowest chlorogenic acid content was observed in SR at 1.511 ± 0.055 mg/g (Figure 7).

### 3.5. Fourier Transform Near-Infrared Spectrometry (FT-NIR) Analysis

The FT-NIR spectra showed some degree of similarity in the chemical composition of the different *A. africana* samples (Figure 8). The highest degree of similarity in the chemical composition was observed among the leaf samples (WL, IL, and SL), which formed up to eight peaks between 9000 and 4000 cm^−1^ (Figure 8).

The root samples (SR and MR) had peaks similar to those of the leaf samples, except between 5000 and 4000 cm^−1^ wavenumbers (Figure 8). Unlike the rest of the samples, the spectrum of CA exhibited a peak at 5100 cm^−1^ (Figure 7). Ward's algorithm-based sample clustering showed the closest homogeneity (0.35) between IL and SL (Figure 8). IR and SR also had a close similarity, with a small heterogeneity value of 0.57 (Figure 8). The highest dissimilarity was recorded between CA and the root samples (IR and SR), with a heterogeneity value of 1.45 (Figure 8).

## 4. Discussion

Although *A. africana* has been studied extensively, there have been few studies on the antioxidant properties of the plant. Most of the previous studies are centered on the antioxidant activities of the plant leaves without exploring other plant parts/tissues [12, 27, 30, 31]. The antioxidant properties of natural products have been widely investigated using DPPH assays [32]. The DPPH antioxidant test demonstrated the ability of a test sample to scavenge free radicals [32]. The assay is based on the reduction of DPPH (colored free radical) methanolic solution by the free radical scavenging action of bioactive compounds or test samples [32]. The DPPH free radical scavenging test on *A. africana* indicated that all the investigated tissues possessed antioxidant properties. Previous studies on *A. africana* leaves have also reported their antioxidant potential [12, 27, 30].

The antioxidant activity of the plant tissues is largely attributed to the presence of bioactive polyphenols, which also possess antimicrobial and anti-inflammatory properties [32, 33]. A number of studies have demonstrated a positive correlation between the polyphenol content of plant samples and their antioxidant capacities [32, 34]. Similarly, our study clearly shows that the higher the total phenolic and flavonoid content in the tissues, the higher the antioxidant activity. Thus, IR, with the highest total phenolic, flavonoid, and chlorogenic acid content, displayed the highest DPPH free radical scavenging capacity and the lowest IC_50_ value. In contrast, SR had the lowest polyphenolic content and exhibited the lowest antioxidant activity. Polyphenols are abundant in *A. africana* [5, 12] as confirmed by our study and may be the main contributor to the antioxidant potential exhibited by its tissues. In a previous study by Niyonizigiye et al. [12], the highest total phenolic and flavonoid content in *A. africana* leaves was 76.61 ± 3.90 mg GAE/g and 62.71 ± 2.10 mg quercetin equivalent (QE)/g, respectively. These values were obtained through heating and agitation extraction techniques. The total phenolic and flavonoid content in all the leaf samples in our study was higher than that seen in the samples of Niyonizigiye et al. [12]. This disparity could be attributed to the differences in extraction technique and the environment since the *A. africana* samples in the two studies were obtained from different geographical regions.

Chlorogenic acid, a phenolic compound and well-known antioxidant [9, 35], was shown in this study to be present in all *A. africana* tissues, with the highest concentration being observed in IR. IR also had the highest antioxidant potential, as exhibited by high DPPH inhibition comparable to the standard antioxidant, gallic acid, and the lowest IC_50_ value (27.25 ± 5.028 *μ*g/mL) among all *A. africana* tissues. The antioxidant properties of the samples were positively correlated with chlorogenic acid content in the sample tissues, except for SL. This indicates that although chlorogenic acid may contribute to the antioxidant capacity of *A. africana* tissues, it is not the main contributor. Rather, it is a part of a large group of polyphenolic compounds present in *A. africana* tissues. In contrast to our observations, there are plant species of medicinal value, for which the antioxidant capacity of the tissues is dependent mainly on chlorogenic acid content [35, 36]. Wu [36] showed that the antioxidant capacity of *Flos Lonicerae* is dependent on its chlorogenic acid content. In his study, Wu [36] demonstrated that *F. Lonicerae* samples with higher chlorogenic acid content exhibited higher efficiency in scavenging DPPH radicals and reducing Fe^3+^ to Fe^2+^. Tomac et al. [35] demonstrated that the antioxidant activity of coffee beans is positively correlated with their chlorogenic acid content. In their study, Tomac et al. [35] compared the antioxidant activity of coffee brands and their chlorogenic acid content. In the same study, Tomac et al. [35] further demonstrated that the mechanism of action of chlorogenic acid as an antioxidant was the direct scavenging of hydroxyl radicals (OH^−^) and direct chemical reactions between chlorogenic acid and the radicals formed from DNA during nucleic acid damage. The antioxidant property of *A. africana* tissues is possibly due to the total phenolic and total flavonoid content in the plant tissues.

The difference in antioxidant activities of the different parts of *A. africana* could be attributed to the difference in the concentration of antioxidant content, mainly total phenolic and flavonoid content in these plant parts. Similarly, Feduraev et al. [37] demonstrated in their study that the antioxidant activities of different parts of *Rumex crispus* L. and *R. obtusifolius* differed from each other. They attributed these differences to the varying phenolic content in the different plant parts. Secondary metabolite content in plant organs of different species varies depending on the developmental stage of the plant and environmental conditions [38, 39]. In our study, IR had the highest concentration of polyphenolic compounds (total phenolic and total flavonoid content), giving it the highest antioxidant capacity, while SR had the lowest polyphenolic content and exhibited the lowest antioxidant activity.

In comparison to a previous antioxidant study on *A. africana*, Johnson et al. [27] revealed that the plant leaf extract had an IC_50_ value of 95.50 *μ*g/mL. This value did not differ much from the IC_50_ values of *A. africana* leaf extracts in our study, which were 99.08 ± 4.483 *μ*g/mL (WL), 124 ± 14.994 *μ*g/mL (SL), and 128 ± 4.606 *μ*g/mL (IL). The minor difference between the IC_50_ value of WL and the IC_50_ value of the leaf extract from the previous study could be attributed to the difference in extracting solvents ([27] used methanol), while the relatively large differences between the IC_50_ value of the leaf extract from the previous study and the IC_50_ values of SL and IL could be due to differences in plant developmental stages, in addition to the extraction solvents used. Unlike in our study, Niyonizigiye et al. [12] obtained a very large DPPH antioxidant activity for *A. africana* ethanolic leaf extract (IC_50_ value: 3 ± 0.03 mg/mL). This difference could be attributed chiefly to the difference in extraction techniques since the green extraction technique was used in the previous study. This difference could also be attributed to differences in the geographical regions from which the plant leaf samples were collected. Guimarães et al. [38] emphasize that the environment influences the secondary metabolite content in plants and thus their activity.

Through scientific studies, calli obtained from various plant tissues have been demonstrated to possess various secondary metabolites and potent biological activity, including antioxidant potential. These plants include *Artemisia amygdalina* [40], *Harpagophytum procumbens* [41], *Vigna unguiculata* [42], *Randia echinocarpa* [43], and *Oroxylum indicum* [44]. Based on this background, we generated calli from *A. africana* leaf explants and used them as part of our study material. *A. africana* calli had good antioxidant activity, with an IC_50_ value of 96.08 ± 4.144 *μ*g/mL. The antioxidant potency of calli from other plants species has also been reported previously, including *H. procumbens* (IC_50_ = 46.74–163.66 *μ*g/mL) [41], *Inula crithmoides* (IC_50_ = 0.09–10.2 mg/mL) [45], and *Justicia gendarussa* (IC_50_ = 15.81–40.75 mg/mL) [46]. The differences observed in the antioxidant activities of the calli are due to varying media and hormonal combinations, explant parts, calli culture duration, and plant species [41, 45, 46].

The FT-NIR technique, known to be a fingerprint technique, captures chemical data in relation to C-H, S-H, N-H, and O-H bonds in the sample [47]. Infrared spectrometry provides valuable information for medicinal plant analysis and quantification of chemical content [48, 49]. The phytochemical content of plant tissues that exhibit antioxidant properties contributes to the NIR spectra [47, 48]. FT-NIR spectra have been used in many studies for the assessment of antioxidant chemical constituents in several plants [47, 48, 50].

The FT-NIR spectral peaks from 4200 to 4900 cm^−1^ are assigned to combination (stretching and deformation) modes due to C-H and O-H groups that belong to phenolic rings [48, 50]. The FT-NIR spectra in our study showed three prominent peaks for all the *A. africana* plant samples within these wavenumbers except for SR, indicating the absence of an antioxidant phenolic phytochemical compound in SR at 4336 cm^−1^, which possibly contributed to its low antioxidizing property in comparison to other *A. africana* samples. The peaks at intervals 5050–5200 cm^−1^ are associated with the combination modes of the O-H group in phenols and the corresponding aromatic ring-related vibrations [48]. Spectral features from 5400–6000 cm^−1^ are due to the first overtones of C-H stretching modes from the corresponding aromatic rings [48, 51]. The spectral peaks from 6050–7200 cm^−1^ are due to second overtones due to C=O stretching in flavonols [50] and O-H combinations in phenols [51]. As shown in the FT-NIR spectra of all the samples, there is a close similarity in the groups of antioxidant chemical compounds present in the *A. africana* samples. The difference in antioxidant abilities could be attributed to the differences in the relative quantities of the antioxidant chemical constituents in the samples, as indicated by the differences in their absorbance.

## 5. Conclusion

The antioxidant activity of *A. africana* tissues was positively correlated with the total phenolic and flavonoid content in the samples. *A. africana in vitro* regenerated roots (IR) had the highest total phenolic content (167.84 ± 1.057 mg GAE/g), total flavonoid content (135.06 ± 0.786 mg RUE/g), and chlorogenic acid content (5.23 ± 0.298 mg/g) and the highest antioxidant capacity, with the lowest IC_50_ value of 27.25 ± 5.028 *μ*g/mL. In contrast, SR had the lowest polyphenolic content and the lowest antioxidant potential. The antioxidant activities of all analyzed *A. africana* tissues varied significantly. Although chlorogenic acid, an important antioxidant phytochemical compound, is present in a number of plants, to the best of our knowledge, this is the first report of this compound in *A. africana* callus (CA) and root tissues. Our study reports, for the first time, the antioxidant activities of *A. africana* callus and roots (*in vitro* and *ex vitro*). IR, CA, and WL tissues of *A. africana* could be valuable natural sources of antioxidants that could be further exploited for the development of useful pharmaceutical products including anxiolytic drugs, given the fact that these tissues are rich in flavonoids and chlorogenic acid that are known to possess anxiolytic effects. We recommend further screening and isolation of the phytochemical constituents responsible for the high antioxidant activities of *A. africana* plant tissues, especially in *in vitro* regenerated roots, wild leaves, and calli.

## Figures and Tables

**Figure 1:** Chemical structure of chlorogenic acid.

**Figure 2:** *Aspilia africana* callus generated from leaf explants. (a) Callus in Petri dish. (b) Callus nature and structure.

**Figure 3:** DPPH antioxidant activities of *A. africana* samples and gallic acid. Values are presented as means ± standard deviation. Same letters are not significantly different by Tukey's test and *p*=0.05.

**Figure 4:** DPPH antioxidant activities of *A. africana* samples and gallic acid. Values are presented as means ± standard deviation. Same letters are not significantly different by Tukey's test and *p*=0.05.

**Figure 5:** Total phenolic and flavonoid contents in *A. africana* samples. (a) Total phenolic contents. (b) Total flavonoid contents. Values are presented as means ± standard deviation. Same letters are not significantly different by Tukey' s test and *p*=0.05.

**Figure 6:** Comparative chromatograms of the different samples of *A. africana* at ultraviolet (UV) detection wavelength of 200–400 nm.

**Figure 7:** Chlorogenic acid contents in different samples of *A. africana* samples. Values are presented as means ± standard deviation. Same letters are not significantly different by Tukey's test and *p*=0.05.

**Figure 8:** (a) FT-NIR spectra for *A. africana* samples. (b) Dendogram of *A. africana* samples analyzed from FT-NIR.

## Data Availability

The data used to support the findings of this study are available from the corresponding author upon request.
